# Use of Medicinal Plants for Respiratory Diseases in Bahawalpur, Pakistan

This article has been retracted.

**DOI:** 10.1155/2021/5578914

**Published:** 2021-04-04

**Authors:** Sadia Afzal, Hafiz Ishfaq Ahmad, Abdul Jabbar, Mahmoud M. Tolba, Sameh AbouZid, Nimra Irm, Farheen Zulfiqar, Muhammad Zahid Iqbal, Shoaib Ahmad, Zubair Aslam

**Affiliations:** ^1^Department of Botany, Faculty of Life Science, Women University Multan, Punjab, Pakistan; ^2^Department of Animal Breeding and Genetics, University of Veterinary and Animal Science, Ravi Campus Pattoki Punjab, Pakistan; ^3^Department of Clinical Medicine, Faculty of Veterinary Science, University of Veterinary and Animal Sciences, Lahore Punjab, Pakistan; ^4^Pharmaceutical Division, Ministry of Health and Population, Faiyum, Egypt; ^5^Department of Pharmacognosy, Faculty of Pharmacy, Heliopolis University for Sustainable Development, Egypt; ^6^Department of Food Science and Human Nutrition, Faculty of Biosciences, University of Veterinary and Animal Sciences, Lahore Punjab, Pakistan; ^7^Faisalabad Medical University, Faisalabad, Pakistan; ^8^Punjab Medical College, Faisalabad, Pakistan; ^9^Department of Agronomy, University of Agriculture, Faisalabad, Pakistan

## Abstract

The most common ethnomedicinal plants being effective in respiratory disorders were studied for the first time in Bahawalpur District. The herbal medication represents a low-cost treatment for the local community. There is a need for documenting the traditional uses of plants for further investigation of bioactive compounds. Using a qualitative approach, the ethnobotanical data was collected from the district of Bahawalpur, Pakistan, from February 2018 to February 2020 through semistructured interviews with the local people and traditional healers. The quantitative analysis included use value, informant consensus factor, family importance value, and relative frequency citation. A total of 20 indigenous plants belonging to 17 families were documented from 185 informants. These plants were claimed to be used for the treatment of 10 respiratory ailments. The plant habit, part of the plant used, and mode of preparation were standardized for authentication. The herbs are the most used life form (55%), while trees and shrubs are also used. Leaves dominate with high use value (47.62%) followed by fruit, stem, flower, and other parts of plants. For the preparation of traditional remedies, decoction (76.19%) and extract (71.43%) are common preparation methods. However, other methods of paste infusion, powder juice, and ash are used to a lower extent. The plants with higher use value are *Glycyrrhiza glabra*, *Acacia arabica*, and *Mentha piperita*; these have significant potential therapeutic activity for respiratory disease. The ethnomedicinal importance of plants against respiratory diseases used by the local population (traditional healers) is the commercial availability of the herbal product. It is a first-time study in this area to fill the gap between traditional practices and synthetic medicine to screen out the phytochemical and pharmacological properties of plants that have a highly futuristic use value to develop antibiotic drug with least side effects by using sustainable methods.

## 1. Introduction

The ethnobotanical importance of medicinal plants predominantly serves to maintain public health from an era of time in many cultures and traditions around the world [1–3]. It is noteworthy to say that the World Health Organization (WHO) stated that 80% of the global population is nutritionally dependent upon plants as a cure for primary health. Additionally, about 11% of essential drugs are originated from plants as phytotherapeutic agents [4]. Therefore, to explore the usage of medicinal plants in the treatment of disease, the researchers gained significant knowledge many years ago [5]. The emerging importance of ethnic usage of medical treatment caused the side effects of allopathic medicine and their cost and unavailability of biomedical treatment due to some factors that were seriously urgent to the local community for the indigenous plant [6].

The geographical position of Pakistan makes this region supplemented with a diversity of medicinal plants used by the indigenous people for the medical care of their animals [7, 8]. The majority of the population is living in rural areas, their source of income is based on agriculture, and their low economic livelihood is dependent on ethnomedicinal plants [9]. Therefore, local people use plant-based remedies using different parts of plants in the traditional form of commercially available herbal products [10]. The medicinal plant is locality matter as it is reported that about 90% of plant species are used by the natives [11].

Many significant respiratory diseases contain upper respiratory tract infection and lower respiratory infection causing asthma, bronchitis, common cold, cough, pneumonia, and whooping cough [12]. The respiratory disorder counted to 2.2 million resulting in deaths every year; therefore, in the treatment of acute infection of the respiratory tract, it exceeds a high cost of 20 billion [13]. Bahawalpur is an area with high temperature where a great range of flora exists with dust storm in summer. A high temperature where a great range of flora exists with dust storm in summer is considered a significant factor for ethnobotanical study [14]. The traditional remedies regarding respiratory diseases for human health care are widespread in this area where people rely more on medicinal plants than synthetic medicine [15]. Contextually, many plants from different families are used from one generation to another to cure cough, asthma, respiratory tract infection, and pneumonia by the indigenous population [16]. Due to the reliability of some definite phytochemicals, the plants are exploited for an extended period conventionally go over for curing diverse ailments [17]. Vast medicinal plants have naturally diverse benefits for mankind as they are very useful against respiratory disease worldwide and in other areas of Pakistan [12, 16]. Plants contain external and internal secreting secondary metabolites, such as phenol, tannins, alkaloid, steroid, resins, and gum related to the antimicrobials associated with antimicrobials [17, 18] and antibacterial [19]. Prospectively, the future must satisfy the therapeutic need for more researches on plants to emphasize the use of medicinal plants in primary health needs [20]. Therefore, the objective of this study was to document the most common medicinal plants used for respiratory disorders, which is done for the first time in this region. Furthermore, it is essential to compile indigenous knowledge of the native area by conducting studies on the pharmacological and phytochemical screening of plant species in order to certify their use in treating various ailments, as well as educating rural people about sustainable plant use and conservation.

## 2. Methods

### 2.1. Study Area

Southern Punjab is a lower area of Punjab, where Bahawalpur lies at (29°24′0^″^N, 71°41′0^″^E) covering an area of 24,830 km^2^ [21]. The population of this division is about 11,464,031, which was estimated in the 2017 census [22]. The Bahawalpur District has a large geographical area, which contains six tehsils Bahawalpur Saddar, Bahawalpur City, Khairpur Tamewali, Yazman, Hasilpur, and Ahmedpur East [15] (Figure 1). A river and well-irrigated canal system are the main water sources of this region, while annual rainfall fluctuates from 90 to 200 millimeters. Cholistan Desert is situated in the south of the city, which expands to the Indo Pak border, containing diversified flora and fauna [14]. It is the southeastern part of the Punjab, where the summer is very hot with dust storms in May and June, while the winter is cold. In the desert where the most essential wildlife is a national park away from the richness of wildlife habitat, ethnobotanical studies are the most important for medicinal plant researches [23].

### 2.2. Data Collection

The ethnomedicinal study of plants for respiratory disorders is undertaken by a structured questionnaire from the population living in the district of Bahawalpur from February 2018 to February 2020, keeping in view the rules of documentation of the ethnobotanical data [24]. For collecting the data of ethnomedicinal plants and the significance of this region, the open-ended and close-ended interviews [25] were conducted on plant locality, the local name of the plant, parts of the plant used, the method used in the preparation, and the plant forms with their usage. To select the informant for indigenous knowledge, a different category was used in which area-wise information was collected from the different age groups in which gender, qualification, income, and experience were considered to analyze the usage of the plant concerning traditional medicine for respiratory diseases. The use of the same species by the informants was characterized and accordingly assessed [26]. On the other side, interviews were also conducted with the 28 traditional healers to peruse medicinal plants as commercial products. All the data obtained from 185 informants and traditional healers were compiled to analyze the locals' use of the medicinal plants.

#### 2.2.1. Demographic Characteristics of Informants

The demographic features of local informants were determined by a questionnaire designed as per the rule of the ethnomedicinal survey. A total of 185 informants were involved in the current study; 139 males were interviewed at their workplace, and 64 females were interviewed at houses through face-to-face conversation. Most of the informants were shopkeepers, farmers, laymen, gardeners, teachers, and housewives. To collect the traditional knowledge regarding medicinal plants, the informants above 60 years were prioritized. The very significant information about the use of medicinal plants in their products was taken from traditional health practitioners through an interview. The questionnaire was also used. Many studies of the ethnomedicinal use of plants have been testified worldwide along with Pakistan [27] and Turkey [28].

#### 2.2.2. Plant Collection and Identification

The traditionally useful plants in respiratory diseases by the natives of Bahawalpur were collected from the area: dried, pressed, and mounted on the herbarium sheet. For the authentication of the plant name index and the list of the plant, http://www.ipni.org and http://www.theplantlist.org were used, respectively, and for the taxonomic verification of the plant, http://www.ars-grin.gov/cgi-bin/npgs/html/queries.pl was used. All the herbarium plants were accompanied by data such as family, their scientific name, local name, life form, part of the plant used, and the association of disease with the plant. Identification and voucher specimen were according to the Flora of China, Scopus, Flora Iranica, Web of Science, and Google scholar and the flora of Punjab [29] and the flora of West Pakistan and Kashmir for the vascular plants [30].

### 2.3. The Quantitative Study of Ethnobotanical Plants

To analyze the quantitative research of the ethnobotanical plants, there are different quantitative directories: use value (UV), informant's consensus factor (ICF), relative frequency citation (RFC), and family importance value (FIV).

#### 2.3.1. Use Value (UV)

This is a method that shows the relative significance of the medicinal plants used by the locals of the studied area. For the standard approach to evaluate a plant's UV, a specific protocol was given by [31]

(1) $$\begin{array}{c} \text{UV}=\sum \;\frac{U}{N}, \end{array}$$

where the informant's numbers are represented by “*N*” which specifies the use of plant species. Its value shows the user report of a specific plant but does not indicate the multiple benefits of a plant.

### 2.4. Informant's Consensus Factor (ICF)

It is the value that refers to the consumption of medicinal plants and analyzes the disease cured by adapted methods. Therefore, the respiratory disorder is sorted into different categories. To calculate the ICF value, the formula is given as

(2) $$\begin{array}{c} \text{ICF}=\frac{N_{\text{ur}-}N_{t}}{N_{\text{ur}-}1}. \end{array}$$

For each category of diseases, the user report (UR) number is indicated by “*N*_ur_” while species of medicinal plant use are represented by “*N*_t_” [32]. To prove the authenticity of locals, the data for the use of medicinal plant range from 0 to 1.00 in which the greater value expresses a high consumption of a medical plant, while the low value tells that the informants rarely use the medicinal plant species.

#### 2.4.1. Relative Frequency Citation (RFC)

The traditional significant value of a plant species in its native area (RFC value) of each species was calculated by respondents that mention the use of specific medicinal plants (FC) by the whole number of informants (*N*) in the survey. The formula is given as [33]

(3) $$\begin{array}{c} \text{RFC}=\frac{\text{FC}}{N}. \end{array}$$

#### 2.4.2. Family Importance Value (FIV)

It is the quantitative measure to analyze the important value of the family and is described by the informants. It is calculated by using this formula:

(4) $$\begin{array}{c} \text{FIV}=\frac{\text{fc}}{n}\times 100, \end{array}$$

where it is the percentage of informant's report for a family of the plant to which it belongs.

## 3. Results and Discussion

### 3.1. Medicinal Plant Documentation and Ethnodemography of the Inhabitants

The most common 21 medicinal plants, belonging to 17 families, are used by indigenous people for 11 associated respiratory diseases. A survey was conducted by 185 informants interviewed; it was classified into different classes of demographic characters shown in Table 1.

The medicinal plants are mostly used to cure respiratory diseases giving designated information as presented in Table 2. The males—75% informants—were interviewed, and 25% of females were included in the survey. The demographic characters are designed in such a way that it showed the experience of the informant with plant species so that traditional healers were also included in studies where 65% have 2–5-year experience; those having 5-10-year experience are 35%, while the most reported locals are under the age of 61-75 (35.1%) followed by the age of 46-60 (30.8%) and 30-45 (21%), and the least are those with age above 75 years. In this study, it is clearer that respiratory disorders prevail more in illiterate people, which is 27%.

### 3.2. Medicinal Plant and Indigenous Experience

The 21 species of medicinal plants that were most recorded have been used for different respiratory diseases (Table 2). These plants belong to 17 different families: *Lamiaceae* (3 species), *Boraginaceae*, and *Zingiberaceae* (2 species), while others reported only one species used by indigenous people. The life form of the plant is very significant because it specifies the environmental condition of the region (Bahawalpur).  Figure 2 shows that herbaceous plants (52.38%) are more common and trees (23.8%) are followed by shrubs (19.10%). The parts of the plants were leaves (47.62%), fruits (33.33), and stem, roots, flower, seed, and bark which were also used to some extent (Figure 3). In ethnobotanical preparation, the leaves were used, so their collection does not impact the life cycle of plants [34]. The leaves are more tolerable for the local plants regarding other life forms of plants or entire plants. The plant's mode of usage depends upon the part of plant use that is delicate, soft, and hard [12]. According to the life form and plant part used in the crude preparation for respiratory disease, many traditional recipes are made with or without a subsidiary substance: decoction (71.4%), extract (66.7%), infusion, paste (38.1%), and powder (33.3%), and least mode of preparations that are made contains juice and ash (14.3%) (Figure 2). The traditional healer role for practice is that they use two or more plant mixes with some other ingredients: water, milk, essential oils, honey, and butter. The most used preparation is a decoction; it is prepared by boiling the plant part in water so that the required amount is obtained. Mostly, the administered dose is internal in this disease, but its external use is also preferred in the form of a paste. The dose and mode of administration to each patient are according to the physical condition and stage of the disease.

### 3.3. Therapeutic Significance

According to the survey from the region of Bahawalpur, the respiratory disease is categorized into 10 disorders (Figure 4). In this region, the most reported diseases in regard to plants are cough (10 species), asthma (8 species), bronchitis (5 species), influenza (4 species), sore throat and respiratory disorder (3 species), and pneumonia and tuberculosis (2 species). Other species are also significant in dry and whooping cough.

### 3.4. The Quantitative Study of Ethnorespiratory Information

#### 3.4.1. The Family Importance Value (FIV)

The family importance value (FIV) indicates the family significance in the region used by the informants, in which the reported dominant family is *Zingiberaceae* with FIV (8.11), followed by *Lamiaceae* (10.27), *Solanaceae* (7.7), *Violaceae and Apiaceae* (6.5), *Anacardiaceae* (5.9), and *Mimosaceae* (5.4), and the families with least FIV are *Acanthaceae and Boraginaceae* (4.86), *Malvaceae* (4.3), and *Arecaceae* (3.78), followed by *Rhamnaceae* (1.6) and *Amaranthaceae* (0.54). This result is shown in Figure 5.

#### 3.4.2. Relative Frequency Citation (RFC)

From different localities of Bahawalpur, the most used medicinal plant for respiratory ailments by the informants shows the RFC value. The highest value shows the highest consumption of medicinal plants including *Zingiber officinale*, *Mentha piperita* and *Withania somnifera* (0.08), and *Mangifera indica*, *Glycyrrhiza glabra*, *Viola odorata*, and *Foeniculum vulgare* (0.06), while the medicinal plant with regard to respiratory disease has low RFC, but their other therapeutic indication has significant value. These are *Justicia adhatoda*, *Ficus religiosa*, *Acacia arabica*, and *Onosma bracteatum* having an RFC value of 0.05.

*Zingiber officinale* is a herb used for cold, cough, throat infection, and influenza where an underground stem is used to make juice and a paste is made by grinding, infusion, and extraction. *Mentha piperita* is a common plant in which leaves and the stem are used to make juice, paste infusion, and extract in water. It is mainly helpful to treat cough, sore throat, and influenza. *Withania somnifera* is a small plant, commonly known as Ashwagandha; its delicate roots make decoction and extracts to treat asthma and bronchitis. Its use in a commercial product for these diseases indicates its significance. *Mangifera indica* is a perennial tree whose bark and leaves are used to treat the sore throat by making juice and paste by crushing the leaves, infusion; bark extract is also made for crude preparation. *Glycyrrhiza glabra* is a small herb plant where the plant's roots are used to make the decoction, paste, and extract helpful in curing asthma, cough, and pneumonia. *Viola odorata* is a common herb commonly known as *Banafsha.* This region is used in traditional remedies for cough and other respiratory disorders by making decoction and extract of stem and root. The decoction, the seeds of *Foeniculum vulgare*, is used to treat cold and cough, while extract and paste of the stem and leaves are consumed for respiratory disorders. *Justicia adhatoda* is a shrub plant that is considered important to cure asthma and cough by preparing extract, paste, powder, decoction, and ash, which is also prepared for tuberculosis and sore throat.

#### 3.4.3. User Value (UV)

The relative importance of medicinal plants by quantitative analysis in a population is known as the plant's user value (UV). The plants with high UV are *Acacia Arabica* (0.91), *Mentha piperita* (0.9), which is contrary to the study conducted in Gujranwala Pakistan, *Glycyrrhiza glabra* (0.89), *Withania somnifera* (0.87), *Mangifera indica* (0.86), *Viola odorata* (0.85), and *Achyranthes aspera* (0.7) [35]. The plants with the highest UV are popular among the indigenous people of Bahawalpur District for respiratory diseases. *Acacia arabica* has antibacterial properties [36], which effectively treats the association of bronchitis, colds, and tonsillitis with respiratory diseases by using pods and leaves to make a decoction and a paste of leaves. *Achyranthes aspera* with a high UV value indicates its extensive use for asthma, bronchitis, cold, cough, and pneumonia in the Bahawalpur. It has been used by making decoction, powder, and extract for asthma. In addition, paste and ash are also used. The plants show their less use by the population due to minimum knowledge and exposure of plant with the natives of the region Bahawalpur. The medicinal plant with lower user value is *Ficus religiosa* (0.68), *Phoenix dactylifera* (0.59), *Curcuma longa* (0.57), *Hyssopus officinalis* (0.5), and *Onosma bracteatum* (0.32). The plant's availability makes a medicinal plant achieving its highest and low user value.

#### 3.4.4. Informant Consensus Factor (ICF)

To analyze medicinal plants important for a disease used by the informant, the usage report is valuable to categorize respiratory disease into ten diseases. The cough is reported for 95.24% plant species by 66 users, followed by cold. Around 85.71% of medicinal plants have been used for asthma, and after that, plants recorded for sore throat (76.19%), bronchitis (66.67%), whooping cough (61.9%), influenza (52.38%), respiratory disorder (47.62%), pneumonia (42.86%), and tuberculosis (33.33%). The study shows that cough and cold are the most prevailing diseases in this area. The same results for disease regarding plants have been described in northern Pakistan [16].

### 3.5. The Medicinal Plant Available in Commercial Products

To confirm the ethnorespiratory plant significance, the market survey of herbal medicine as drugs for the usage of plants was conducted to treat respiratory disease. It is reported that five plants among the 20 plants belong to commercial treatment as respiratory disease drugs; local healers used these plants with other substituents in commercially available plants with a great source of income for the local community and traditional healer. The data of plants used commercially is shown in (Table 3).

### 3.6. Comparative Study of Plants in Respiratory Disease

The ethnorespiratory plant analysis was compared in other studies in many regions of Pakistan and our neighboring countries to conform to the stated data. The comparison of this study showed that the plants reported in the Bahawalpur region were also used for respiratory diseases in another region (Table 4).

The study at west Azerbaijan shows the respiratory disease cured by traditional medicinal plants showing a similar study. Some 20 plants used in treating disease, the species of *Mentha*, have the same uses as our study [12]. The study of ethnobotanical plants in *manisia* where the plant has similar uses and modes of preparation through *Glycyrrhiza glabra*, but there is a contrast in the use of plants *Mentha x piperita* L and *Foeniculum vulgare* Mill. So, there is the novelty of the use of plants against respiratory disorder [37].

The area of Bahawalpur, Pakistan, was reported with 123 plants out of these 7 species, which uses *Achyranthes aspera*, *Mangifera indica*, *Phoenix dactylifera*, *Mentha longifolia*, *Acacia nilotica*, *Withania somnifera*, and *Phyla nodiflora*, with properties to cure respiratory diseases [38].

A similar study in the Northern region shows 120 plants with 5 plants having comparable uses and modes of preparation including *Acacia nilotica* (L.), *Glycyrrhiza glabra* L. *Justicia adhatoda*, *Achyranthes aspera*, *Abelmoschus esculentus* (L.) [27] studied 85 medicinal plants *Mentha longifolia*, *Achyranthes aspera*, *Withania somnifera*, and *Ficus religiosa* tally with plants used in the present study while some plants having dissimilar use are *Mangifera indica* and *Acacia arabica* [16, 39]. A study in Uganda, 2 plants out of 88 plants, *Mangifera indica L* and *Achyranthes* aspera L, are used for respiratory disease, but its use in tuberculosis is more emphasized [40].

A previous study contains 129 plants in which 4 plants with have same use including *Justicia adhatoda*, *Achyranthes aspera*, *Withania somnifera*, and *Ficus religiosa* are included, but 2 plants have dissimilar use and these plants are *Mangifera indica* and *Acacia nilotica* [41]. 384 medicinal plants from which 8 plants have been studied with similar use. The plant's similar use for respiratory diseases is *Glycyrrhiza glabra*, *Onosma bracteatum*, *Zingiber officinalis*, *Viola odorata* L., *Mangifera indica*, *Ficus religiosa* L, *Phoenix dactylifera*, and *Phyla nodiflora* [42].

It was reported, in India, that 57 medicinal plants belong to 37 families and 53 genera [43]. The plants, used for respiratory disease, are *Acacia nilotica (L.) Curcuma longa*, *Withania somnifera*, and *Zingiber officinale* while the plants *Achyranthes aspera*, *Ficus religiosa*, and *Mangifera indica* have dissimilar use with the present study. 100 plants were studied and no one has similar uses, but these plants have other expectorant and diuretic viz. *Acacia nilotica*, *Achyranthes aspera*, and *Mentha longifolia* [44].

## 4. Conclusion

This survey examines the most common uses of medicinal plants against respiratory diseases in the district of Bahawalpur, Pakistan. The indigenous people of this region use the native plants to cure their respiratory diseases because of synergistic and preventive causes. The most common plants belong to different families like *Lamiaceae*, *Fabaceae*, *Papilionaceae*, *Anacardiaceae*, *Zingiberaceae*, *Solanaceae*, and *Arecaceae*, which can cause associated respiratory symptoms: cough, asthma, bronchitis, and pulmonary infection. Traditional healers also use the plants, but the commercial manufacturer's used plants and other plants in herbal medication help ease the dilemmas of respiratory disorders. The exploration of ethnomedicinal information is necessary to value the traditional use of medicinal plants by the local community. Thus, bioassay and frequency of plant-related drugs can be executed relationally. The present study is an enduring survey supporting the prospect by documenting the traditional knowledge of indigenous plants of this area and raising the significance of old practices for treatment. As a contextual recommendation, the need for an hour is to establish research to screen out the important phytochemicals in plants and develop the antibiotics by using these plants, which have resistance against bacteria and have the least side effect on the human body. Contextually, this survey is to fill up the gaps between the traditional usage of plants and pharmacological studies of respiratory disorders to document ethnomedicinal data in a meaningful way. A conventional method of collecting the parts of plants is recommended so that its life cycle is not disturbed as well as the survival of endangered species of plants is not affected.

## Figures and Tables

**Figure 1:** Study area map—Bahawalpur District, Pakistan.

**Figure 2:** Mode of preparation used in the respiratory treatment and life form of a plant.

**Figure 3:** Plant part used for respiratory disease.

**Figure 4:** FCI value of plant against respiratory diseases.

**Figure 5:** Family importance value of plants.

**Table 1:** Demographic knowledge of informants in the current study.

Variable	Demographic variants	Number	Percentage (%)
Gender	Male	139	75
	Female	64	35
Plant species			
Age	30-45	39	21
	46-60	57	30.8
	61-75	65	35.1
	>75	24	12.9
Informants	Locals	157	84.8
	Traditional healers	28	15.1
Education	Illiterate	50	27
	Elementary	28	15.1
	Secondary	20	10.8
	Undergraduate	48	25.9
	Graduate	39	21
Experience of TH	2-5 years	18	65
	5-10 years	10	35

**Table 2:** Most common medicinal plant species of Bahawalpur District with their use values, relative frequency citation, and family importance value.

Name of plant	Family name	Common name	Plant part used	Preparation method	Life form	Therapeutic effects	UR	FC	UV	RFC	FIV
*Justicia adhatoda* BP01	*Acanthaceae*	Malabar nut	Leaves	Extract, paste, ash, powder, decoction	Shrub	Asthma, cough, sore throat, tuberculosis	2	9	0.67	0.05	4.86
*Achyranthes aspera* BP02	*Amaranthaceae*	Puthkanda	Root	Decoction, powder, extract, paste, ash	Herb	Asthma, bronchitis, cold, cough, pneumonia	4	1	0.7	0.01	0.54
*Mangifera indica* BP03	*Anacardiaceae*	Mango	Bark, leaves	Juice, paste infusion, extract	Tree	Sore throat	1	11	0.86	0.06	5.95
*Foeniculum vulgare* BP04	*Apiaceae*	Fennel	Seeds and leaves, flower	Decoction, powder, extract, paste, ash	Herb	Respiratory disorder cold, cough	4	12	0.65	0.06	6.49
*Phoenix dactylifera* BP05	*Arecaceae*	Date palm	Fruit	Decoction, extract, powder	Tree	Bronchial infection	2	7	0.59	0.04	3.78
*Cordia obliqua* BP06	*Boraginaceae*	Lasora	Fruit, leaves	Powder, extract	Tree	Dry cough, tuberculosis	3	7	0.61	0.04	3.78
*Onosma bracteatum* BP07	*Boraginaceae*	Gaozaban	Fruit, leaves	Extract, decoction, infusion	Herb	Respiratory tract infection, influenza	4	9	0.32	0.05	4.86
*Glycyrrhiza glabra* BP08	*Fabaceae*	Liquorice	Roots	Decoction, extract, paste	Herb	Asthma, cough, pneumonia	2	12	0.89	0.06	6.49
*Thymus vulgaris* BP09	*Lamiaceae*	Thyme	Leaves, flower	Decoction, powder, extract, paste, ash	Shrub	Bronchitis, whooping cough	3	8	0.54	0.04	4.32
*Mentha piperita* BP10	*Lamiaceae*	Peppermint	Leaves, stem	Juice, paste infusion, extract	Herb	Cough, sore throat, influenza	2	14	0.9	0.08	7.57
*Hyssopus officinalis* BP11	*Lamiaceae*	Zoofa	Herb	Decoction, extract, powder	Shrub	Cough	2	5	0.5	0.03	2.7
*Abelmoschus esculentus* L. BP12	*Malvaceae*	Okra	Seed fruit	Powder	Herb	Asthma	2	8	0.63	0.04	4.32
*Acacia arabica* BP13	*Mimosaceae*	Kiker	Fruit and leaves	Decoction, extract, powder	Tree	Bronchitis, cold tonsillitis	4	10	0.91	0.05	5.41
*Ficus religiosa* BP14	*Papilionaceae*	Peepal	Fruit, leaves	Extract, paste, ash	Tree	Asthma, tuberculosis	1	9	0.68	0.05	4.86
*Ziziphus vulgaris* BP15	*Rhamnaceae*	Anab	Fruit, leaves	Extract, decoction, infusion	Shrub	Cough and cold, influenza	3	3	0.29	0.02	1.62
*Withania somnifera* BP16	*Solanaceae*	Ashwagandha	Roots	Decoction extract	Herb	Asthma, bronchitis	4	14	0.87	0.08	7.57
*Phyla nodiflora* BP17	*Verbenaceae*	Cape weed	Whole plant	Infusion	Herb	Asthma, influenza	2	6	0.57	0.03	3.24
*Viola odorata* BP18	*Violaceae*	Banafsha	Stem, root	Extract, decoction, infusion	Herb	Respiratory disorders	3	12	0.85	0.06	6.49
*Curcuma longa* BP19	*Zingiberaceae*	Turmeric	Underground stem	Extract, decoction, infusion	Herb	Pulmonary infection, tuberculosis	4	6	0.57	0.03	3.24
*Zingiber officinale* BP20	*Zingiberaceae*	Ginger	Stem	Juice, paste infusion, extract	Herb	Cold, cough and throat infection, influenza	2	15	0.91	0.08	8.11

**Table 3:** Commercial availability of plants in herbal products.

Commercial products	Treatment associated	Major plants included in the herbal product	References
Suduri	Bronchitis	*Ocimum basilicum*, *Adhatoda vasica*	[45]
Infuza	Asthma	*Glycyrrhiza glabra*	[45]
Joshina	Bronchitis	*Ziziphus sativa*, *Viola odorata*, *Adhatoda vasica*	[45]
Sharbat Banafsha	Cough	*Viola odorata*	[46]
Shaafi Joshanda	Cough	*Adhatoda vasica*, *Viola odorata*, *Foeniculum vulgare*	[45]
Linkus	Cough	*Adhatoda vasica*, *Foeniculum vulgare*, *Viola odorata*	[45]
Joshinda	Bronchitis	*Ocimum basilicum*, *Onosma bracteatum*, *Ziziphus sativa*, *Viola odorata*	[45]
Johar Joshanda	Cough	*Ocimum basilicum*, *Viola odorata*	[46]
Corezcol	Expectorant	*Mentha arvensis*, *Adhatoda vasica*	[46]

**Table 4:** Comparison of similarities and differences between the study area and neighboring regions.

Area	References	No. of species	Plants with similar use	Plants with different use	Similarity ratio
Urmia	[12]	20	1	0	0
Turkey	[45]	137	1	2	1.46
Bahawalpur, Pakistan	[46]	123	7	0	0
Gallies, Northern Pakistan	[16]	120	5	0	0
Hafizabad, Pakistan	[27]	85	4	2	2.35
Uganda	[37]	88	2	0	0
Pakistan	[38]	384	8	0	0
Lahore, Pakistan	[39]	129	4	2	1.55
Uttar Pradesh, India	[40]	57	4	3	5.26
Swat, Pakistan	[41]	100	0	3	3

## Data Availability

The numerical data used to support the findings of this study are available from the corresponding author upon request.
